The article "Application of Uncertainty Thought Environment in Judicial Adjudication Based on Cognitive Psychology" was retracted in 2023. Reasons: signs of a paper mill; suspected computer-generated content; unreliable results or conclusions; concerns about the data.

# Application of Uncertainty Thought Environment in Judicial Adjudication Based on Cognitive Psychology

**DOI:** 10.1155/2022/1088046

**Published:** 2022-09-06

**Authors:** Yongchao Li

**Affiliations:** Zhengzhou University School of Law, Zhengzhou 450001, China

## Abstract

The uncertainty of judicial decision-making has a deep and extensive theoretical foundation. Theoretical analysis starts with a reflection on legal rationalism that challenges the legal certainty before delving deeply into the case's facts and the entire legal system. In light of this, this paper explores a novel approach to enhance the reasoning mechanism of trial documents from the viewpoint of modern cognitive psychology, concentrating on the parties' and the public's cognitive processes to justice. It is suggested to use an inert hierarchical multilabel classification algorithm. In order to predict the category of invisible examples, the extended multilabel training set is first searched for adjacent samples of invisible examples, and the classification weight and confidence of each category are then determined in accordance with these adjacent samples. The group of invisible examples is then anticipated. Experimental comparison demonstrates that this algorithm outperforms other prediction techniques; the macro accuracy, macro recall, and macro *F*1 of this method are, respectively, 0.896, 0.871, and 0.814. It has some advantages in many multilabel evaluation indexes when compared to other multilabel algorithms.

## 1. Introduction

Currently, China has undergone numerous judicial reforms, all of which have their roots in the judge's decisions. With high-level design, China has begun a new phase of judicial reform, but there are still many challenges and obstacles in the way of actual judicial operations. The actions taken by judicial operators to take into account rationality have been affirmed but also come under heavy criticism and doubt given the current climate of China's judicial system, which promotes positive justice, strong mediation, and attention to the unity of legal effect and social effect. There are two types of uncertainty: objective uncertainty and subjective uncertainty. The event's outcome is uncertain because there are many possible ways for it to follow its own motion law, which is the definition of objective uncertainty [1]. There must be some objective standards to judge whether justice is done fairly or not, even though this is a highly subjective assessment and the solution is a very difficult one. Judges may encounter a variety of challenges and difficulties during the fact-finding, legal discovery, and decision-making processes. As a result, judges' decisions become increasingly ambiguous, drawing the interest of academic circles.

The article "Application of Uncertainty Thought Environment in Judicial Adjudication Based on Cognitive Psychology" was retracted in 2023. Reasons: signs of a paper mill; suspected computer-generated content; unreliable results or conclusions; concerns about the data.

The objective of justice is to render a fair and reasonable decision, and the presumption to achieve this objective is that the judge must stand in an impartial and objective position to learn the facts of the case and must be just to apply the rules of legal judgement. Although the Anglo-American legal evidence system recognises the concept of judicial cognition, judges in countries with civil law systems always introduce prior knowledge into their core testimony [2, 3]. It is now common practise in all nations to use probability theory and psychological information system theory to examine the evidence of judgements due to the development of modern cognitive psychology and the new school of evidence law. Without the state, law, and government, people can achieve complete material and spiritual freedom. Because of this, the author chose to interpret Kennedy's understanding of political law and the judicial reasoning process from the perspective of Kennedy's critical legal ideas, particularly from the perspective of the uncertainty of judicial decisions, and analyse its rationality and irrationality. Extensive research was carried on the validation and comprehension of judgement uncertainty. The author's ultimate goal is to develop a rational understanding of the pertinent issues of judicial adjudication through a combination of research and demonstration. This understanding will serve as a useful guide for developing a national rule of law and judicial reform.

Sentence documents are texts, which fall under the category of unstructured data, so the general classification algorithm cannot directly handle them, which makes them one of the challenges in automatically determining the law that applies to a case. Automatically determining the relevant legal issues in a case is a multilabel classification problem as opposed to the traditional classification problem in DM (data mining) [4] because a case frequently can be applied to multiple legal provisions. A framework describes a group of words with a similar cognitive structure and a dominant semantic role. It also establishes complex static and dynamic relationships between frameworks, involving both concrete facts and abstract ideas. And explain how over time, concepts are related by static entities. Judicial decisions are inferences from observed evidence to assumptions that infer causes from observed evidence, in order to maintain neutrality between probability and explanatory inference based on inference.

The innovation of this paper is as follows:

1. We define the assumption in the judicial field as the preliminary speculation or prejudice caused by the judge's processing of information through an intuitive mechanism based on legal prediction, especially at the stage when the pretrial information is insufficient. Reveal the reasons for the uncertainty of judicial decisions, that is, the uncertainty of legal norms and legal reasoning process.
2. In order to identify the applicable law of the case more effectively and automatically, it is necessary to analyze the characteristics of the problem more deeply. One of the research contents of this work is to extract the factual description of the case and its applicable legal provisions from the sentencing documents, and structure them to form the feature vectors and category labels of sample cases.

The article "Application of Uncertainty Thought Environment in Judicial Adjudication Based on Cognitive Psychology" was retracted in 2023. Reasons: signs of a paper mill; suspected computer-generated content; unreliable results or conclusions; concerns about the data.

## 2. Related Work

### 2.1. Research Status of Domain Cognitive Bias in Psychology

In social interactions, cognitive deviation is a frequent psychological occurrence. People first became interested in it as a psychological phenomenon, and as time went on, more and more fields of study began to be included in the research. Different disciplines have different perspectives on cognitive bias when it comes to definition. As cognitive subjects must be aware of cognitive objects, which are impersonal entities, different cognitive environments will have an impact on their cognitive outcomes. In order to fully define cognitive bias, these three components are necessary.

Mann et al. analyzed several common cognitive bias types and combined them with school education, which has a very important academic value [5]. Garip et al. studied the influence of cognitive bias on management decisions [6]. Kang et al. found that compared with healthy people without anxiety disorder, anxiety disorder patients have a greater and more lasting influence on some negative suggestive words, indicating that the influence of cognitive bias on anxiety of anxiety disorder patients is not instantaneous or one-way factorial [7]. Lees argues that the study of cognitive bias should not stay on the phenomenon, but should pay attention to the mechanism of cognitive bias [8].

Starting from the specific problems faced by judges exercising judicial power, Lekakis summarized the uncertainty of judicial decisions by analyzing the micro judicial process of finding out facts, finding out laws, and making decisions that must be solved in the judicial process [9]. Frailing et al. found that the dilemma encountered by the theory of admissibility of judicial decisions lies in the fact that it provides a legitimate reason for transforming heterogeneous factors outside the law, such as public opinion, into a standard ruling within the legal scope. This runs counter to the concept of “taking law as the criterion” [10].

The article "Application of Uncertainty Thought Environment in Judicial Adjudication Based on Cognitive Psychology" was retracted in 2023. Reasons: signs of a paper mill; suspected computer-generated content; unreliable results or conclusions; concerns about the data.

### 2.2. Research on Text Mining Technology

An important step of automatic identification of applicable law of a case is to use text mining technology to process the text of the case facts and get the structured representation of the case facts. The objects of text mining are massive, heterogeneous and distributed texts, and the content of texts is the natural language used by human beings, which lacks the semantics understandable by computers. Therefore, the main problem faced by text mining is how to represent the text in a reasonable way, so that it can contain enough information to fully reflect the characteristics of the text, without being too complicated for the learning algorithm to handle.

Zou et al. discussed the views of Bayesian doctrine and Bayesian skepticism, thinking and waiting for the probability analysis of reasoning to realize the fact finding [11]. Al-Luwaici et al. believe that the first step of the jury's factual verdict is to code the evaluation of the evidence [12]. In the process of constructive explanation of his holistic law theory, Zhang et al. put forward the theory of understanding coherence, pointing out that coherence is the value that holistic law should have [13]. Kumar et al. used autocorrelation and Fourier transform techniques to detect the periodicity of moving objects, and then used hierarchical clustering algorithm to count the periodicity of moving objects [14]. Sering et al. put forward a method to determine the number of clusters in *K*-means algorithm. When the minimum number of clusters is greater than 2, *K*-means algorithm is used to evaluate the clustering effect of different clusters, and the number of clusters with the best clustering result is obtained [15].

Law and Ghosh determined the category of a document according to the probability that words of related categories appear in a document. Because this method is too simple and mechanical, the classification effect is not very good [16]. The upsampling method proposed by Borhani et al. mainly adopts the idea of interpolation and takes the data between a few samples and one of its adjacent samples as a new sample of a few classes. Over-fitting in oversampling [17]. Charte et al. proposed a new feature selection algorithm, which uses Hellinger distance, mainly because Hellinger distance is not affected by uneven data distribution. The larger the Hellinger distance of the feature, the stronger the classification ability of the feature, so the more representative it is, the better the effect of this new method is [18].

## 3. Methodology

### 3.1. Psychological Structure Observation of Judicial Cognition in Civil Litigation

The assumption of justice is in the blind spot of the dual analysis framework of formal rationality and substantive rationality. Some guilty verdicts are the compound product of substantive conviction conditions and guilty premises, and it is impossible to achieve zero innocence. It can only be done by limiting the influence of judicial presumptions for the sake of formal rationality and conscious equal protection of civil rights. It includes a system for intuitive processing and a mechanism for rational analysis as a cognitive processing channel linking outside stimuli and learned responses. Irrational intuitive systems typically present a streamlined cognitive model, so they typically take the lead. The disjunction between facts and existence, however, is a feature of the judicial trial process, and the trial theories advanced by the legal community are challenged by a number of challenging issues, including numerous theoretical monologues.

The article "Application of Uncertainty Thought Environment in Judicial Adjudication Based on Cognitive Psychology" was retracted in 2023. Reasons: signs of a paper mill; suspected computer-generated content; unreliable results or conclusions; concerns about the data.

The pursuit of justice is a challenging political, social, and psychological issue. Personal experiences and sentiments play a significant role in how the public and the parties assess the fairness of a court, a location, or even a nation. There is a lot of uncertainty and it varies from person to person and place to place. A person's current knowledge, experience, and cognitive make-up will have a significant impact on his or her psychological activities and outward behaviours, while his or her internal psychological activities regulate and control all of their outward behaviours, including their actions, speech, and behaviour generation.

The process by which the human brain encodes, stores, and retrieves input data is known as memory. In judicial decision-making, it is crucial, and procedural knowledge is even more crucial. However, most of the information that regular people know about legal rulings falls under the category of declarative knowledge. Therefore, the satisfaction of litigants can only be significantly increased by further promoting judicial openness, ensuring procedural fairness, guaranteeing litigant rights in accordance with the law, respecting citizens' democratic rights, and establishing a judicial system free from barriers.

Human cognition is limited in scope. When faced with a large amount of information, we automatically select the information that is more significant and appealing while ignoring the rest. If the judge only considers the personalities, appearance, educational attainment, and other characteristics of the parties without taking into account the legal relationship itself, the judge's final judgement is inevitably going to contain a lot of subjective information. In order for the judge's judgement to naturally connect with the process and shape the judgement outcome, the plan in the judge's head will give the judge the context and process of the entire development of the case. While information about a person's behaviour can assist us in establishing and contacting the causal relationship of behaviour, information about a specific person can aid us in partially understanding the entirety of the situation. The regulation of legal cognitive deviation primarily begins with increasing the accuracy of judges' intuitive perception because there are restrictions on how to extract legal provisions. Several factors show how this intuitive perception affects the accuracy of legal knowledge.

The article "Application of Uncertainty Thought Environment in Judicial Adjudication Based on Cognitive Psychology" was retracted in 2023. Reasons: signs of a paper mill; suspected computer-generated content; unreliable results or conclusions; concerns about the data.

The analysis and gathering of intelligence information is hampered by the fact that information and data from all walks of life are largely autonomous and independent of one another. All types of information can be integrated, and this requirement for data collection can be eliminated or weakened. The design of the data warehouse is analysis-oriented; it starts with the most fundamental theme, continually creates new themes, enhances existing themes, and finally creates a theme-oriented analysis environment. By knowing the data in the initial database system and the data in the subject of the data warehouse to be built, a data-driven system has the advantage of making full use of the existing system and reducing the workload of building the system. The application model of behavioral data warehouse consists of four parts, as shown in Figure 1.

Multidimensional data [19] and data warehouse make up the central data warehouse. After being extracted, transformed, and cleaned, the source data is loaded into the behaviour information data store. For ease of analysis, the data is centralised, cleaned, and converted in the data warehouse. Users are connected to data warehouse and multidimensional database through the service layer, which has the data warehouse and DM technology at its core. Users are shown the results of the analysis by the visualisation layer, which can also re-analyze the data shown and use it to create the final analysis report.

Data is usually represented by attributes. For example, people can be represented by attributes such as height, weight, skin color, occupation, etc., Generally, the noise processing in data cleaning adopts the method of averaging the measured values. Data integration is used to reduce the redundancy of attributes and calculate whether attributes are redundant. Pearson product moment coefficient can be used, which is expressed as follows:

(1) $$\begin{array}{c} r_{A,B}=\frac{\sum_{i=1}^{n}\left(a_{i}-\bar{A}\right)\left(b_{i}-\bar{B}\right)}{N\sigma_{A}\sigma_{B}}=\frac{\sum_{i=1}^{N}\left(a_{i}b_{i}\right)-N\bar{AB}}{N\sigma_{A}\sigma_{B}}, \end{array}$$

where *r*_*A*,*B*_ ∈ [−1,1], *a*_*i*_, *b*_*i*_ are the values of the object on the attribute *A*, *B*, $\bar{A}$ is the average value of the attribute *A*, $\bar{B}$ is the average value of the attribute *B*, *σ*_*A*_ is the standard deviation of the attribute *A*, and *σ*_*B*_ is the standard deviation of the attribute *B*.

The article "Application of Uncertainty Thought Environment in Judicial Adjudication Based on Cognitive Psychology" was retracted in 2023. Reasons: signs of a paper mill; suspected computer-generated content; unreliable results or conclusions; concerns about the data.

There is a query operation set *Q*={*Q*_1_,…, *Q*_*n*_}, and the query frequencies are *f*_*Q*_1__,…, *f*_*Q*_*n*__, respectively. For materialized view set *M*={*V*_1_,…, *V*_*k*_}, the total query cost is

(2) $$\begin{array}{c} QE\left(E\right)=\sum_{i=1}^{n}f_{Q_{i}}*E_{Q_{i}}\left(M\right), \end{array}$$

where *E*_*Q*_*i*__(*M*) is the cost of calculating query *M* using materialized view set *Q*_*i*_.

Mahalanobis distance represents the covariance distance of data. It is an effective method to calculate the similarity of two unknown sample sets.

(3) $$\begin{array}{c} d\left(x_{i},x_{j}\right)=\left(x_{i},x_{j}\right){\sum^{-1}\left(x_{i},x_{j}\right)}^{T}, \end{array}$$

where ∑ is the covariance matrix.

The logical model design of the data warehouse needs to roughly estimate the data magnitude of the future data warehouse, and then, determine the relatively reasonable data granularity according to this rough estimated value. Simple estimation method of data magnitude in data warehouse is

(4) $$\begin{array}{c} \alpha \times \left(\sum_{i=1}^{N}\left(S_{i}+K_{i}\right)\times L_{\max}^{i}\times T\right)∼\alpha \times \left(\sum_{i=1}^{N}\left(S_{i}+K_{i}\right)\times L_{\min}^{i}\times T\right), \end{array}$$

where *N* is the number of tables in the conceptual model; *S*_*i*_ is the size of the table; *K*_*i*_ is the key size of the table; *L*_max_is the maximum number of records and the minimum number of records is *L*_min_ per unit time; *T* is the period that data exists in the data warehouse; *α* usually takes 1.2–2.

### 3.2. Multilabel Classification of Uncertainty in Judicial Decisions

Some critics have effectively applied the principles of cognitive psychology and made empirical research on the intuitive processing mechanism in judicial process. They pointed out that in the case of insufficient information and uncertain judgement, intuition provided the premise for legal reasoning by introducing legal provisions and preliminary training. Conclusion logical automatic intuition can also bypass the cognitive process and reach a conclusion quickly. As a knowledge structure system organized by judges in advance, legal foresight affects judges' perception and attention to laws and facts, and constitutes judges' cognitive framework and vision. Unless key new evidence is found or stronger reasoning appears in the trial, the judge will not overturn the prebuilt hypothesis.

The article "Application of Uncertainty Thought Environment in Judicial Adjudication Based on Cognitive Psychology" was retracted in 2023. Reasons: signs of a paper mill; suspected computer-generated content; unreliable results or conclusions; concerns about the data.

Critical jurisprudence is an approach to research, a methodology, or a method rather than a distinct and organised philosophy. The fact that there are differences should cause us to reflect more on how various cultural and social factors influence our judgement and how to formulate the final judgement. The interests of the majority of groups can currently be used to determine the dominant legal ideology in China. Chinese legal thought successfully combines normative and descriptive elements. It addresses the inherent requirements of socialist rule of law, such as people's democratic ideas, legal beliefs, Marxist jurisprudence, and socialist moral values, in an open and inclusive structure.

To achieve an orderly, stable, harmonious, and effective legal system, it is necessary to control the uncertain legal factors within a reasonable range. The traditional, well-known spirit of reason and legal certainty is also a myth and cult that borders on the insane. In this case, a large number of witnesses lie under oath or are obstinately biased against the prosecution, and some of them are ignorant of the facts of the case or have false memories. There is no room for improvement if the law is wholly fixed as of the date of creation. Due to the diversity of the cases, this allows the law to be insufficient. As a result, when making decisions, judges constantly seek a foothold in their own value resources. The value judgement itself is frequently neither good nor bad; rather, it merely reflects personal preferences.

The power structure, the evolution of the law, and citizen morality will all be impacted by the use of algorithms in the legal system. Therefore, rule-making necessitates both predictive capability and decision-making cost, and decision-makers must take into account potential future behaviours as much as possible. A tree-like class hierarchy must be supported by the corresponding multilabel hierarchical classification algorithm, which is an unbound leaf node prediction algorithm used to address the issue of automatically identifying applicable rules in cases. Any node in the class hierarchy can correspond to the predicted class labels.

In the traditional single label classification task, based on the assumption that all labels in the label set are independent of each other, an instance is only associated with a certain label in the label set [20]. In the actual classification task, multiple labels can describe an object, so as to classify it more accurately. The process of defining multilabel classification tasks is as follows:

(5) $$\begin{array}{c} \overset{⟶}{y_{x}}\left(l_{i}\right)=\arg\max_{b\in \left\{0,1\right\}}P\left(H_{b}^{l_{i}}\right)P\left(E_{\overset{⟶}{C_{x}}\left(l_{i}\right)}^{l_{i}}|H_{b}^{l_{i}}\right), \end{array}$$

where $\overset{⟶}{C_{x}}\left(l_{i}\right)$ in the formula is an element in the vector $\overset{⟶}{C_{x}}$ of 1 × *q*, which indicates how many of the *k* nearest neighbors of the sample instance contain this label for a label *l*_*i*_.

The article "Application of Uncertainty Thought Environment in Judicial Adjudication Based on Cognitive Psychology" was retracted in 2023. Reasons: signs of a paper mill; suspected computer-generated content; unreliable results or conclusions; concerns about the data.

At the same time, the calculation method of label distribution of documents becomes

(6) $$\begin{array}{c} R_{d}=\left(\theta_{d}^{\prime }+\theta_{d}^{\prime \prime }\right)\times \eta \times \varphi_{t}. \end{array}$$

When the model is stable, count the count values of the topic-tag pairs of words to obtain *T* × *C* matrix, and superimpose the matrix on the topic dimension to obtain *C*-dimensional tag vector, which represents the statistical values of the tags assigned to the words in document *d*.

In order to solve the problem of automatic identification of applicable laws of cases, this paper proposes an inert multilabel hierarchical classification algorithm. Lazy learning methods can well support incremental learning. When a new training sample is added, it only needs to be merged with the stored training sample, so that the new training sample can participate in the prediction process and get a new training sample. The framework of the algorithm is shown in Figure 2.

In the prediction stage, the algorithm finds the *k* nearest neighbor samples from the multilabel extended training set and calculates the confidence *k* instances that unseen instance belongs to each category according to the nearest classification weight and neighbor samples of each category, and then classify the invisible instances into the appropriate classes according to the threshold decision. Through the transformation of training set, the hierarchical structure of tag space is considered as a whole, so that the prediction results can directly meet the hierarchical constraints, without additional correction process.

For sample (*x*_*i*_, *y*_*i*_)((*x*_*i*_, *Y*_*i*_) ∈ *N*(*x*)), assuming that it has *n* category labels, the classification weight of the sample for category *y*_*j*_ is

(7) $$\begin{array}{c} w_{ij}=\left\{\begin{array}{cc} \frac{1}{n}, & y_{j}\in Y_{i},\\ 0, & y_{j}\notin Y_{i}. \end{array}\right. \end{array}$$

If the sample has a category label, the corresponding weight is set to 1/*n*, otherwise it is 0. Choosing 1/*n* as the sample weight is calculated by entropy maximization.

When the document *d* is predicted, the count values of 〈*t*_1_, *t*_2_, *c*〉 pairs of words are counted, and the matrix of *T*_1_ × *T*_2_ × *C* is obtained. Firstly, the matrix is superimposed on the *T*_1_ dimension, and then, on the *T*_2_ dimension to obtain the label vector of the *c* dimension, which represents the label count value of the words in the document *d*. Then, the label distribution of the document was calculated:

(8) $$\begin{array}{c} \theta^{d}=\frac{N_{c}^{d}}{\sum_{c=1}^{d}N_{c}^{d}}. \end{array}$$

The diagonal elements of the matrix *M* form a *C*-dimensional vector *N*, and the *i*th element of the vector represents the total value of the label *j* count. Then, the probability of label *j* appearing when label *i* appears can be calculated by

(9) $$\begin{array}{c} p\left(C_{i}|C_{j}\right)=\frac{M_{ij}}{N_{j}}. \end{array}$$

If *p*(*C*_*i*_*|C*_*j*_)=1, it means that label *i* is the parent node of label *j*.

The article "Application of Uncertainty Thought Environment in Judicial Adjudication Based on Cognitive Psychology" was retracted in 2023. Reasons: signs of a paper mill; suspected computer-generated content; unreliable results or conclusions; concerns about the data.

The negative correlation labels of all the labels of sample *x*_*i*_ are obtained by using the label information of neighboring samples, and if the label *l*_*j*_=0 of sample *x*_*i*_ is trained, then *N*_*ij*_=0; otherwise, the calculation formula of *N*_*ij*_ is as follows:

(10) $$\begin{array}{c} N_{ij}=\arg\max_{\notin Y_{i}:k\neq j}P\left(l_{j}=1|l_{k}=0,N\left(x_{i}\right)\right), \end{array}$$

where *l*_*j*_ represents the *j*th tag in the training set and *l*_*k*_ tag represents a tag that does not belong to the sample *x*_*i*_. Considering that a tag may also affect a tag when it doesn't appear, the input in the algorithm is the same as that in constructing the positive correlation matrix *P* of the sample tag pair.

## 4. Experiment and Results

In this chapter, the effectiveness of this method in evaluating the workload of judges is tested through experiments. Compared with other traditional algorithms, this method not only improves the number of iterations, but also improves the clustering quality. In this paper, the clustering quality is judged by the contour coefficient, and the clustering result with the highest contour coefficient is considered as the best clustering result. The data used in the experiment is the data retrieved from judicial investigation. The number of test samples is 600, and the *k* value when the average contour coefficient is the largest is taken as the optimal number of groups. The following Figure 3 shows the relationship between the number of groups and the average contour coefficient.

Through the experiment, it can be concluded that when *k* takes different values, the contour coefficient is different, and when *k*=50, the clustering effect is the best.  Table 1 shows the number of clusters with the best clustering effect and the corresponding average contour coefficient values.

The article "Application of Uncertainty Thought Environment in Judicial Adjudication Based on Cognitive Psychology" was retracted in 2023. Reasons: signs of a paper mill; suspected computer-generated content; unreliable results or conclusions; concerns about the data.

It can be seen that the method in this work has significantly improved the quality of clustering. Although it takes time and space, it has achieved good clustering results, and the algorithm is still desirable. The traditional algorithm not only has some blindness in choosing *k* value in experiments, but also has some limitations in dealing with different data sets. Using the algorithm in this document, in step 1, the size of the general moving average window is 8, and the number of groups is *k*=5; in step 2, if the trend similarity threshold is selected as 1, the different projection time series of each stage will be the numbers shown in Figure 4.

The majority of unqualified objects will be eliminated after the first two rounds of screening, so in the third round of screening, it is still necessary to calculate the temporary distance between the two time-series because the candidate objects are already large, reduction in amplitude. It will take much less time to complete this process as a result. However, it is much more accurate to define the trend similarity of time series and the similarity of Euclidean distance than it is to define the similarity of Euclidean distance directly from the perspective of wave pattern.

Figure 5 shows the prediction accuracy values of the three algorithms under different neighbor node values. It can be seen from the Figure 5 that the hybrid recommendation algorithm is more accurate than the original collaborative algorithm. The prediction accuracy increases with the increase of the number of neighbors. When the number of neighbors is 48, a better accuracy can be achieved. The accuracy of this algorithm is 0.85. When the number of nodes exceeds 48, the accuracy is not improved.

Dynamic scalability, or how to add new algorithms without affecting existing DM algorithms, must also be taken into account in the implementation process in addition to providing DM services to the outside world. The coupling between submodules should be minimised during design, and users should only need to call a specific interface without being aware of the implementation's details. It realises data storage and offers data upload and download in data management. It also provides a parallel algorithm library that can run on the Hadoop platform. It offers data on task status and node status for resource management. Because our method doesn't consider the dependency between tags, the uneven distribution among high-level tags is difficult to detect and deal with, so the classification of topic and tag level is poor; The feedback in our method follows the label and inherent hierarchy between topics, but is not supervised by probability; in order to verify the scalability of the model, five indexes of the dataset with three-tier label structure are compared in the experiment. The results are summarized in Figure 6.

The article "Application of Uncertainty Thought Environment in Judicial Adjudication Based on Cognitive Psychology" was retracted in 2023. Reasons: signs of a paper mill; suspected computer-generated content; unreliable results or conclusions; concerns about the data.

It can be seen that the average results of this method are superior to other discipline models in all five groups of measurement indexes, which shows that this method still has advantages in extending the dataset to three-tier label structure. The number of datasets in the negative model is too small, and this small amount of data is concentrated in the training set with poor classification effect, which makes the prediction accuracy of the model poor. The experimental results show that the classification accuracy of multilabel documents can be improved by selecting appropriate segmentation ratio and fusion method of positive and negative samples for dataset features. Here, the parallel collaborative filtering algorithm based on Map Reduce is tested.  Figure 7 shows the acceleration of the parallel collaborative filtering algorithm.

It can be seen from Figure 7 that the enhanced collaborative filtering algorithm based on Map Reduce has a good speed-up ratio. With the increase of the number of nodes, the speed-up ratio gradually increases, but then the speed-up ratio slows down. This is because Hadoop platform interacts between nodes through the network. With the increase of the number of nodes, the communication time between nodes increases, resulting in a slower increase in throttling ratio. It can also be seen from the Figure 7 that the acceleration ratio is directly proportional to the size of the dataset.

Table 2 shows the prediction performance of various algorithms in each macro-average evaluation index. Generally speaking, the method in this paper is obviously superior to the traditional algorithm in macro-average evaluation index.

The comparison of the above experiments shows that the proposed algorithm can achieve better prediction performance than the existing methods. The macro accuracy, macro recall, and macro *F*1 of this method were 0.896, 0.871, and 0.814, respectively. Combined with the characteristics that this document algorithm supports incremental learning, we can use this document algorithm to build an effective and executable automatic identification system for the applicable law of the case.

According to the various ways that people process information, psychologists categorise people's thought processes into left brain and right brain thinking. The use of creative thinking in judicial adjudication is not just a simple grammatical rhetorical device, but rather the collision and integration of adjudicative thinking and popular thinking. It is a method that cannot be disregarded to raise the standard of adjudicative reasoning. The parties and the general public now have higher expectations for judicial justice as a result of the consolidation of court documents and their public dissemination on the Internet, and the court has stricter guidelines for the legal reasoning in court documents. Fundamentally, this is a debate about public perception and judgement thinking. In order to further strengthen the judge's decision-making and public perception, as well as to increase the trial's persuasiveness, it would be wise to strengthen the logic of the supporting documents.

The article "Application of Uncertainty Thought Environment in Judicial Adjudication Based on Cognitive Psychology" was retracted in 2023. Reasons: signs of a paper mill; suspected computer-generated content; unreliable results or conclusions; concerns about the data.

Numerous factors, including logical coherence, morality, and values, affect the judge's decision-making process. Even though logic isn't the only thing that influences how a judgement is made, its importance in this process should not be understated. In a logical sense, it restrains the judiciary, prohibits judicial specialisation, reflects the justice and fairness of the decision, and increases the authority of the court and the law. The legal process is to make a decision in accordance with the established relationship and method, and its particular form is to arrange the competing viewpoints and contentious issues in accordance with the criteria that have been agreed upon by all parties. In contrast, procedural fairness can guarantee convergence and predictability of outcomes in the majority of similar cases. Legal facts can be realised with certainty as long as the impact of legal uncertainty is kept within a reasonable range.

## 5. Conclusions

The certainty and uncertainty of the law are two significant contradictions that, while distinct in the field of law, work in tandem to advance both the development of the law itself and the establishment of the rule of law. Any meaningful knowledge is based on the secondary construction of common sense, so it makes sense that judges make substantive arguments based on common sense assertions and their understanding of meaning, such as experience and ideas. The ability of the verdict to be widely accepted by the parties and the general public following its publication depends on whether or not its language scheme, content scheme, and rhetorical scheme match the existing schemes of the parties and the general public, according to cognitive psychology. In this paper, a multilabel lazy hierarchical classification algorithm is proposed, which can be used for such big and expanding classification problems and is well suited for the automatic identification of case law. Experimental comparison demonstrates that this algorithm outperforms other prediction techniques; the macro accuracy, macro recall, and macro *F*1 of this method are, respectively, 0.896, 0.871, and 0.814. The algorithm suggested in this paper fully takes into account the correlation between tag pairs, including both positive and negative correlation, which helps the classifier perform more accurately in terms of classification.

The article "Application of Uncertainty Thought Environment in Judicial Adjudication Based on Cognitive Psychology" was retracted in 2023. Reasons: signs of a paper mill; suspected computer-generated content; unreliable results or conclusions; concerns about the data.

## Figures and Tables

**Figure 1:** Analysis of the basic architecture of behavioral data warehouse.

**Figure 2:** Algorithm framework.

**Figure 3:** Relationship between clustering number and average contour coefficient.

**Figure 4:** Number of dissimilar time series screened in each stage.

**Figure 5:** Accuracy of three algorithms in different neighbor nodes.

**Figure 6:** Classification result of the data set.

**Figure 7:** Speed-up ratio of parallel collaborative filtering algorithm.

**Table 1:** Experimental results.

Method	Cluster number	Average contour coefficient
[16]	50	0.83
[19]	50	0.862
Methods of this paper	50	0.896

**Table 2:** Performance comparison of hierarchical indexes of algorithms.

Method	Macro accuracy (%)	Macro recall (%)	Macro *F*1 (%)
[16]	0.826	0.801	0.763
[19]	0.833	0.836	0.714
Methods of this paper	0.896	0.871	0.814

## Data Availability

The data used to support the findings of this study are available from the author upon request.
